# *Panax Notoginseng* Saponins Regulate Transforming Growth Factor-*β*1 through MAPK and Snail/TWIST1 Signaling Pathway to Inhibit Epithelial-Mesenchymal Transition of Pulmonary Fibrosis in A549 Cells

**DOI:** 10.1155/2022/3744618

**Published:** 2022-07-12

**Authors:** VietDung Nguyen, Fei Pan, GuangZhong Zhang, Qing Zhang, Yang Lu

**Affiliations:** ^1^Beijing University of Chinese Medicine, Beijing 100029, China; ^2^Beijing Hospital of Traditional Chinese Medicine, Beijing 100010, China

## Abstract

*Panaxnotoginseng* saponins (PNS) is one of the active components of traditional Chinese medicine *Panax notoginseng* which has the function of reducing oxygen consumption, expansion of the cerebrovascular system, and is antithrombotic. PNS also plays a role in the treatment of pulmonary fibrosis. In this study, we found that PNS suppresses fibroblast-like changes in A549 cells through epithelial-mesenchymal transition (EMT). PNS promoted *E-cadherin* (E-cad) in epithelial cells and decreased *Fibronectin* (FN) and *Vimentin* (Vim) expression in myofibroblasts in a dose-dependent manner. Further mechanism studies have shown that PNS inhibits the EMT process by regulating p38, JNK, and Erk signaling factors in the MAPK signaling pathway and then blocking Snail and TWIST1 transcription factors from entering the nucleus. This indicates that PNS can regulate epithelial-mesenchymal transition through MAPK and the Snail/TWIST1 signaling pathway, thereby exerting its antipulmonary fibrosis effect.

## 1. Introduction

Pulmonary fibrosis (PF) is a group of noninfectious and noncancerous respiratory diseases and is the final pathological manifestation of many interstitial lung diseases. PF has extensive extracellular matrix deposition, myofibroblast accumulation, and lung remodeling [1, 2]. Although many studies have focused on patients with PF, the underlying cause of the disease remains unclear. Patients are therefore often diagnosed with idiopathic interstitial pneumonia (IIP), the most common of which is idiopathic pulmonary fibrosis (IPF) [3, 4]. PF usually manifests as exertional dyspnea. With the development of the disease, PF patients will eventually die of respiratory failure. Common clinical symptoms of PF, including fatigue, dry cough, and dyspnea, seriously affect the overall quality of life of the patient [5]. Since there is no treatment to reverse pulmonary fibrosis, slowing disease progression, relieving symptoms, and improving quality of life are the main goals of intervention. The drugs used in the treatment of PF mainly include immunosuppressants, corticosteroids, and antifibrosis drugs, such as Pirfenidone and Nintedanib [6, 7]. However, due to its complex etiology and unclear pathogenesis [8], the efficacy of existing drugs is still not satisfactory. Finding effective new drugs for PF has become a clinical demand and a hot research topic [9].

Epithelial-mesenchymal transition (EMT) is a process in which epithelial cells lose their functions and properties under certain physiological or pathological conditions and transform into mesenchymal cells. Its main biological functions are to make fibroblasts and repair tissue damage caused by wounds and inflammation [10]. EMT plays an important role in embryonic development, chronic inflammation, tissue remodeling, cancer metastasis, and various fibrotic diseases. During EMT, epithelial cells lose their attachment to the basement membrane and acquire a migratory and invasive phenotype. Evidence suggests that EMT promotes the development of pulmonary fibrosis [11]. Among the various stimuli involved in pulmonary fibrosis, transforming Growth Factor-*β*1 (TGF-*β*1) is one of the important factors. It has been proved that TGF-*α*1 can induce EMT and induce signal transduction through classical pathway involving downstream phosphorylation of Smad 2/3 or other pathways, such as Wnt/*β*-catenin signal pathway [12].

*Panax notoginseng* saponins (PNS) are effective medicinal components extracted from *Panax notoginseng*, including a variety of saponin active substances, trace elements, proteins, rich vitamins, and polysaccharides. PNS has the effects of reducing oxygen consumption, dilating cerebral vessels, and it is antithrombotic, anticoagulant, and antifibrotic [13, 14]. Studies on PNS on bleomycin-induced rat IPF have shown that PNS can improve and delay bleomycin-induced pulmonary fibrosis in rats [15]. Additional studies have reported that PNS could improve cardiopulmonary function and inhibit the progression of pulmonary fibrosis through the NF-*κ*B pathway [16].

Mitogen-activated protein kinases (MAPK), also known as serine/threonine protein kinases, can be activated by different extracellular stimuli such as cytokines, neurotransmitters, and hormones. Cell stress and cell adhesion can activate the MAPK signaling pathway, phosphorylate nuclear reverse transcription and regulate the corresponding genes involved in tissue fibrosis. Experiments confirmed that the MAPK signaling pathway is activated in TGF-*β*1-induced pulmonary fibrosis signal transduction [17, 18]. MAPK signaling can inhibit the activity of GSK-3*β* and block the degradation of Snail transcription factor, resulting in its increased accumulation in the nucleus. It was shown that the MAPK pathway can increase the level of Snail, thereby reducing the expression of E-cadherin and promoting the occurrence of EMT [19]. Therefore, our research group intends to establish the A549 cell model to determine whether PNS can inhibit EMT through the MAPK signaling pathway and to further reveal the role and mechanism of PNS in inhibiting pulmonary fibrosis.

## 2. Materials and Methods

### 2.1. Materials

Recombinant human TGF-*β*1 was from PeproTech Inc (Rocky Hill, NJ, USA). Xuesaitong injection (the composition is PNS) was purchased from Harbin Zhenbao Pharmaceutical Co., Ltd. Anti-Fibronectin (15613), anti-E-cadherin (20874), anti-Vimentin (10366), anti-Snail (bs-1371R), and anti-TWIST1 (P106287) were purchased from Proteintech Group Inc. (Campbell Park, Chicago, USA). Antiphospho-p38 (Thr180/Tyr182), anti-p38 (D13E1), antiphospho-JNK (Thr183/Tyr185), anti-JNK (56G8) and antiphospho-Erk (T202/Y204), and anti-Erk (137F5) were purchased from Cell Signaling Technology (Danvers, MA, USA). Inhibitors SB203580 (S1076), PD98059 (S1177), and SP600125 (S1460) were purchased from Selleck Inc (Jin Shan, SH, China).

### 2.2. Cell Culture and Grouping

#### 2.2.1. Cell Culture

Epithelial cells of human lung cancer A549 cell line were purchased from the National Experimental Cell Resource Sharing Platform (Beijing, China). A549 cells were cultured with F-12 medium (containing 100 IU/mL penicillin, 100 mg/L streptomycin and 10% fetal bovine serum) at 37°C in a 5% CO2 incubator. After reaching 80% cell confluence, digested, passaged or related experiments were performed using 0.25% Trypsin.

#### 2.2.2. Establishment of Models and Grouping

A549 cells cultured in vitro were randomized into the control, TGF-*β*1 group and treatment group. The control group was A549 cells + F-12 medium. TGF-*β*1 group was A549 cells + F-12 medium + 10 ng/ml TGF-*β*1. The treatment groups were A549 cells + F-12 medium + PNS concentration with different gradients of 62.5 *μ*g/ml, 125 *μ*g/ml, and 250 *μ*g/ml. The cells were cultured for 72 h.

### 2.3. MTT Cell Viability Assay

Cells were seeded in 96-well plates at a density of 5 × 10^3^ cells/well and incubated overnight. Cells were treated with PNS and PNS + TGF-*β*1 for 72 h. MTT reagent (5 mg/ml) was added to each well and incubated for an additional 4 hours at 37°C. However 100 *μ*L of lysis buffer was added to each well and incubated overnight at room temperature. Finally, the microplate reader was set to detect the optical density (OD) value at 570 nm. The experiments were performed thrice, each in triplicate.

### 2.4. Cell Morphology Observation Experiment

The cells in each well of the 6-well plate were observed and imaged in a visual field magnified 200x using an inverted microscope. Five samples were randomly selected for each group to take photos of, and five random visual fields were counted for each sample for cell morphology detection. Based on a previously established quantitative analysis of cell morphology, the effect of PNS on the morphological structure of A549 cells was tested. Cell roundness was quantified using the image Pro-plus 6.0 software.

### 2.5. Transwell Chemotaxis Assay

The cells were digested with trypsin (0.25%), and the supernatant was discarded. The cell suspension was added without FBS medium to the transformation chamber (100–200 *μ*l/well). The chamber was placed in medium supplemented with 20% FBS. The medium was poured into the cross-well chamber and the bottom of the chamber was wiped with a cotton swab. Placed 4% paraformaldehyde (500 *μ*l/well) into the converter chamber, stained with 0.1% crystal violet solution, and soaked for 30 min. Slices were rinsed twice with distilled water. The chamber was placed on the slices and the migrating cells were visualized by an inverted microscope under the condition of 50x magnification. After incubation at 72 h, cells were stained with crystal violet solution and counted under a microscope for migration. Imagination in a visual field is magnified 100x using an inverted microscope.

### 2.6. Quantitative Real-Time PCR

One-step extraction of total RNA after drug intervention using Trizol. The purity of the RNA was identified and then transcribed backwards onto cDNA. The cDNA was used as a template, and primers of the target genes (FN, Vim, E-cad, Snail, and TWIST1) and internal reference gene (*β*-actin) were added into the reaction system. The reaction conditions were set for PCR amplification of the target gene. There was a linear relationship between the CT value of the template and the number of initial copies of the template. Among them, FN, Vim, E-cad, Snail, TWIST1, *β*-actin, and mRNA full-length PubMed sequence were used as templates, and primers for PCR were designed using Oligo software. A7500 real-time fluorescent quantitative PCR system (Thermo Fisher, Waltham, MA, US) was used. The primer sequences are listed in Table 1.

### 2.7. Western Blot Analysis

The A549 cells were washed twice with PBS, an appropriate amount of cell lysate was added, ice bathed for 30 min, and the supernatant was collected after high-speed centrifugation. The protein concentration was determined by the BCA method, adjusted to the standard concentration, and 10–20 *μ*L samples were taken, respectively. Perform SDS-PAGE electrophoresis and transfer to the PVDF membrane by the semidry transfer method. 5% nonfat milk powder was blocked for 1 h, and primary antibodies were added respectively at the following dilution ratios: *β*-actin, FN, Vim, E-cad, Snail, TWIST1, p-p38, p-JNK, p-Erk, incubated overnight in a 4°C freezer, and then used as antibody Rabbit IgG secondary antibody was incubated at 37°C for 1 h. The membrane was washed with PBST buffer for 10 min × 3 times, and the protein expression on the membrane was observed by the electrophoresis gel imaging analysis system (Tanon, Pujiang High-tech Park, SH, China).

### 2.8. Immunofluorescence Detection

A549 cells were seeded on sterile cover glasses placed on six well slabs. The cells were fixed with 4% paraformaldehyde formaldehyde, infiltrated with 0.1% Triton X-100 for 10 minutes and blocked with 1% bovine serum albumin for 10 minutes. Cells were placed at room temperature and incubated with anti-E-cad antibody, anti-Vim antibody, anti-FN antibody, antiphospho-p38 antibody, antiphospho-JNK antibody, and antiphospho-Erk antibody overnight at 4°C. Cells were washed with PBS and incubated with goat anti-rabbit IgG (A-11010) at room temperature in the dark. Nuclei were counterstained with Hoechst 33342 for 5 min. Cells were fixed with antifade solution and visualized by fluorescence microscopy at 500x magnification.

### 2.9. Statistical Analysis

All statistical analysis was performed utilizing SPSS programming (SPSS 19.0). Comparisons between multiple groups were performed by one-way ANOVA. In the case of homogeneous variance, the LSD method was used to compare the data. When variance between groups was not homogeneous, data were compared using Dunnett's T3 test. *P* < 0.05 was a statistical difference.

## 3. Results

### 3.1. PNS Did Not Significantly Inhibit the A549 Cells

After different concentrations of PNS and PNS + TGF-*β*1 were treated for 72 h, MTT results showed that 31.25∼500 *μ*g/ml PNS and PNS + TGF-*β*1 did not significantly inhibit the A549 cells (Figure 1).

### 3.2. PNS Attenuated the Performance of Pulmonary Fibrosis in the A549 Cell Model

The intervention effect of PNS on the TGF-*β*1-induced pulmonary fibrosis model was observed under an inverted microscope. As shown in Figure 2, TGF-*β*1 showed a significant change in cell morphology from paving stone to spindle shape with a significant decrease in the circularity compared to the control group. Cell circularity was significantly increased in the 125 *μ*g/ml and 250 *μ*g/ml PNS Treatment groups compared to the TGF-*β*1 group. The above experimental results show that PNS can effectively improve and alleviate TGF-*β*1-induced cell fibrosis-like changes while preserving the morphological structure of epithelial cells.

### 3.3. PNS Inhibits Chemotactic Recruitment of Fibrotic Cells

The effect of PNS on the chemotactic activity of A549 cells was measured by transwell. The chemotaxis of cells in the TGF-*β*1 group was higher than that in the control group, as shown in Figure 3, indicating that TGF-*β*1 could facilitate the chemotactic recruitment of A549 cells. However, after PNS treatment at 125 *μ*g/ml and 250 *μ*g/ml concentrations, the cell chemotaxis index was greatly reduced. It was demonstrated that PNS could attenuate the chemotactic activity of TGF-*β*1 on A549 cells, thereby blocking the progression of pulmonary fibrosis.

### 3.4. PNS Can Inhibit the EMT Process by Promoting Epithelial Cell Markers and Reducing the Expression of Mesenchymal Cell Markers

The role and mechanism of PNS in the TGF-*β*1-induced pulmonary fibrosis cell model were investigated by measuring E-cad, FN and Vim. As shown in Figures 4(a) and 4(b), compared with the control group, the mRNA and protein expressions of FN and Vim in the TGF-*β*1 group were increased, while the mRNA and protein expressions of E-cad in the TGF-*β*1 group were decreased, indicating that TGF-*β*1 can significantly mediate the EMT process. Notably, PNS treatment increased the expression of the epithelial cell markers E-cad mRNA and protein, and decreased the expression levels of mesenchymal cell markers FN and Vim mRNA and protein. The results showed that PNS inhibited the occurrence of EMT in a concentration-dependent manner, so the 250 *μ*g/ml treatment group was selected to continue the next experiment. As shown in Figure 4(c), the E-cad fluorescence in the TGF-*β*1 group was significantly weakened, and the E-cad fluorescence expression was enhanced after adding PNS treatment. In addition, the fluorescence of FN and Vim increased significantly in the TGF-*β*1 group, and the fluorescence expression of FN and Vim decreased after adding PNS treatment.

### 3.5. PNS Prevents EMT by Inhibiting TGF-*β*1-Induced MAPK Signaling Pathway

In order to observe the relationship between the induction time of TGF-*β*1 and the expression intensity of the MAKP signaling pathway, we measured the expression levels of p38, p-p38, JNK, p-JNK, Erk, and p-Erk at different times. As shown in Figure 5(a), it was found that p-p38, p-JNK, and p-Erk protein increased most significantly after 72 hours of TGF-*β*1 stimulation, indicating that 72 hours was the best time for TGF-*β*1 to induce the MAPK pathway expression.  Figure 5(b) shows that TGF-*β*1 can increase p-p38, p-JNK, and p-Erk protein. The addition of PNS treatment decreased p-p38, p-JNK, and p-Erk proteins. We confirmed the above results using the immunofluorescence assay. The results in Figure 5(c) indicated that the fluorescence of p-p38, p-JNK, and p-Erk was significantly enhanced in the TGF-*β*1 group, and the fluorescence expression was weakened after adding PNS treatment. To ensure the association between the MAPK signaling pathway and EMT, inhibitors of three signaling factors were added: p38, Erk, and JNK. As shown in Figure 5(d), E-cad was decreased by TGF-*β*1 and restored by MAPK inhibitor. Mesenchymal markers FN and Vim are increased by TGF-*β*1 and decreased by MAPK inhibitor. TGF-*β*1-induced MAPK phosphorylation signaling factors p38, Erk, and JNK were significantly inhibited by the addition of PNS treatment. Treatment with three MAPK signaling factors p38, Erk, and JNK inhibitors was found to be the same as PNS treatment. Prove that PNS can prevent the occurrence of the EMT process through the MAPK signaling pathway.

### 3.6. PNS Can Prevent the Expression of Snail and TWIST1 Induced by TGF-*β*1 While Regulating Snail, and TWIST1 Can Improve the EMT Induced by TGF-*β*1 in A549 Cells

Snail and TWIST1 are classic transcription inhibitors that induce EMT, which regulate the expression of E-cad and Vim. Through this mechanism, they induce the occurrence of EMT in the epithelial-mesenchymal transition. As shown in Figures 6(a) and 6(b), qPCR and Western blotting were performed to examine whether TGF-*β*1 promotes Snail and TWIST1 expression and whether PNS eliminates EMT processes through snail and TWIST1. In these results, Snail and TWIST1 transcripts were upregulated by TGF-*β*1 and inhibited by PNS, SB203580, PD98059, and SP600125. The results in Figure 6(c) demonstrate that PNS, SB203580, PD98059, and SP600125 blocked the action of TGF-*β*1, thereby inhibiting the migration and accumulation of Snail and TWIST1 from the cytoplasm to the nucleus. These data suggest that Snail and TWIST1 are key transcription factors for PNS blockade of EMT.

## 4. Discussion

It was considered many years ago that the pathogenesis of pulmonary fibrosis is the result of progressive inflammation and cell damage leading to the activation and proliferation of lung interstitial cells [20, 21]. However, with the development of medicine, more and more research confirms that inflammation and chronic fibrosis are not necessarily related [22]. Recent research suggests the EMT phenomenon is very closely related to pulmonary fibrosis. EMT reduces E-cad in epithelial cells, increases FN, and Vim in fibroblasts, and promotes fibrotic remodeling [23–25]. Our results suggest that TGF-*β*1 stimulation significantly altered cell morphology from pebbly to spindly and promoted chemotactic recruitment in A549 cells. However, chemotactic recruitment of A549 cells was attenuated after PNS treatment and maintained their original morphology, and PNS increased E-cad expression and decreased FN and Vim expression. Our findings are essentially in line with previous studies, but this study has further explored its mechanism. We studied the effects of PNS on the MAPK signaling pathway and related transcription factors Snail and TWIST1 to explore the deep mechanism of PNS on Pulmonary fibrosis [26, 27]. Overall, this data indicated that PNS could effectively improve and treat pulmonary fibrosis through the MAPK signaling pathway and related transcription factors in an in vitro model.

EMT is a process in which cells with an epithelial phenotype differentiate into a mesenchymal phenotype, and it is involved in physiological processes such as human embryonic development and wound repair. It also plays a key role in human organ fibrosis and tumor pathogenesis. The process of EMT is inseparable from TGF-*β*1. During TGF-*β*1-induced EMT, epithelial cells lose cell-cell connections, induce causing them to isolate from surrounding cells and acquire mesenchymal-like characteristics. TGF-*β*1, a major fibroblast promoter of IPF progression, induces differentiation of lung fibroblasts into myofibroblasts, produces high levels of collagen, and results in loss of lung elasticity and function [28]. TGF-*β*1 can promote or inhibit the growth of epithelial cells and can also participate in the differentiation of alveolar epithelial cells and the activation of fibroblasts [29]. Some researchers have also found that TGF-*β*1 contributes to the disturbance of the lung microenvironment, which leads to the accumulation of a large number of fibroblasts and the deposition of extracellular matrix, accompanied by inflammation and damage to the lung structure, eventually leading to pulmonary fibrosis [30]. TGF-*β*1 could mediate EMT through the classical pathway, bind to the TGF-*β* membrane receptor, and then activate the receptor serine/threonine kinase [29]. Subsequently, Smad is phosphorylated and transferred from the cytoplasm to the nucleus, leading to the activation of the Snail family and the inhibition of E-cad, which ultimately mediates EMT. In addition, TGF-*β*1 also mediates EMT through nonclassical pathways and phosphorylates downstream protein kinase B (AKT) through phosphoinositide-3-kinase (P13K) and MAPK pathways (JNK, p38, Erk), resulting in loss of phosphorylation. Live glycogen synthase kinase 3 (GSK-3B) inhibits Snail phosphorylation and enucleation degradation and increases the level of Snail in the nucleus. Fundamental components of the MAPK signaling pathway are a highly conserved tertiary enzymatic cascade from yeast to humans, including MAP kinase kinase kinase (MKKK), MAP kinase kinase (MKK), and MAPK. These three kinases can be activated in turn and together regulate a variety of important cellular physiological and pathological processes, including cell growth and differentiation [31].

Evidence suggests that EMT is regulated by multiple transcription factors, such as Snail and TWIST1. Snail is an important transcriptional inhibitor regulating E-cad expression in epithelial-mesenchymal transition. The high expression of Snail is a necessary condition for the occurrence of EMT in pulmonary fibrosis. Zhu et al. [32] To study paraquat (PQ) intoxication-induced pulmonary fibrosis and found that hypoxia-inducible factor-1*α* (HIF-1*α*) and EMT are linked to the progression of pulmonary fibrosis. The findings suggest that HIF-1*α* induces EMT by promoting Snail transcription factor, which leads to pulmonary fibrosis. However, TWIST1 is also a critical transcription factor that induces EMT and can regulate the expression of Vim. Mammoto et al. [33] found that vascular remodeling is one of the pathogenesis of pulmonary fibrosis, and they proved that the transcription factor TWIST1 can promote the occurrence of pulmonary fibrosis epithelial-mesenchymal transition. Therefore, regulating the expression of TWIST1 is a curative strategy for pulmonary fibrosis. Taken together, ectopic expression of Snail and TWIST1 may be involved in reducing epithelial cells and increasing mesenchymal cells to induce EMT, ultimately leading to pulmonary fibrosis. Our findings suggest that PNS can effectively inhibit the migration of Snail and TWIST1 from the cytoplasm to the nucleus, preventing EMT and further treating pulmonary fibrosis.

*Panax notoginseng* saponins is one of the main active ingredients of *Panax notoginseng*, a commonly used blood activating herb in Chinese medicine, and has a variety of pharmacological effects, including enhancing immunity, promoting tissue growth, and antitumor effects [34, 35]. In recent years, several research studies have shed light on the significant therapeutic effect of PNS on lung fibrosis. For instance, the mechanism of action of PNS in the treatment of pulmonary fibrosis was studied, and the expression of IL-6 and IL-8 in the PNS group was significantly decreased [16]. They proved that PNS can reduce AST, LDH, CK, IL-6, and IL-8 in rabbit serum by inhibiting the NF-*κ*B signaling pathway and mitigate pulmonary fibrosis. Liu et al. [15] explored the effect of *Panax notoginseng* saponins inhalation solution (TIS) on bleomycin-induced IPF in rats, and found that TIS could improve and delay bleomycin-induced IPF in rats. Our results are consistent with previous studies suggesting that TGF-*β*1 increases FN and Vim expression and decreases E-cad levels. In this study, PNS reversed the progression of pulmonary fibrosis by blocking the expression of transcription factors Snail and TWIST1 through the MAPK signaling pathway and inhibiting epithelial-mesenchymal transition (Figure 7).

## 5. Conclusions

Taken together, our study shows that PNS can improve and treat pulmonary fibrosis by modulating EMT occurrence through MAPK and Snail/TWIST1 signaling pathways. Currently, COVID-19 is spreading around the world, and some patients still have pulmonary fibrosis after being cured [36, 37]. Therefore, finding effective drugs for the treatment of PF has become an urgent need and a research hotspot.

## Figures and Tables

**Figure 1:** Effects of different concentrations of PNS and PNS + TGF-*β*1 on A549 cells proliferation rate. ^*∗*^*P* < 0.05 vs. Control.

**Figure 2:** Comparison of cell morphology and cell circularity in each group (magnification, ×200). vs. control group. ^＃^*P* < 0.01 vs. TGF-*β*1 group.

**Figure 3:** Effects of PNS on the chemotactic activity of pulmonary fibrotic cells by transwell assay (magnification, ×100). ^*∗*^*P* < 0.001 vs. Control group. ^＃^*P* < 0.01. ^＃＃^*P* < 0.001 vs. TGF-*β*1 group.

**Figure 4:** By detecting EMT-related PNS, it was found that PNS could effectively inhibit the occurrence of TGF-*β*1-induced EMT. The gene and protein of E-cad, FN, and Vim were detected by qPCR and Western blotting, respectively (a)-(b). ^*∗*^*P* < 0.05. ^*∗∗*^*P* < 0.01. ^*∗∗∗*^*P* < 0.001 vs. Control group. ^＃^*P* < 0.05. ^＃＃^*P* < 0.01. ^＃＃＃^*P* < 0.001 vs. TGF-*β*1 group. (c) Then immunofluorescence technology was selected to further detect the fluorescence expression levels of EMT signal molecules E-cad, Vim, and FN (magnification, ×500).

**Figure 5:** PNS inhibits epithelial-mesenchymal transition through the MAKP signaling pathway. To study the expression level of the MAPK signal pathway under different time conditions stimulated by TGF-*β*1 (a). ^*∗*^*P* < 0.05. ^*∗∗*^*P* < 0.01. ^*∗∗∗*^*P* < 0.001 vs no TGF-*β*1 added. (b) Next, 72 hours was selected as the stimulation time of TGF-*β*1, and Western blotting was used to detect the protein expression of p38, p-p38, Erk, p-Erk, JNK, and p-JNK related signaling molecules in the MAPK signaling pathway. ^*∗*^*P* < 0.01. ^*∗∗*^*P* < 0.001 vs. Control group. ^＃^*P* < 0.05. ^＃＃^*P* < 0.01. ^＃＃＃^*P* < 0.001 vs. TGF-*β*1 group. (c) Then select immunofluorescence technology to further detect the fluorescence of p-p38, p-Erk, and p-JNK signaling molecules related to the MAPK signaling pathway (magnification, ×500). (d) After adding 3 kinds of MAPK signal pathway inhibitors (SB203580/PD98059/SP600125), Western blotting was used to detect E-cad, FN, and Vim protein related to EMT. ^*∗*^*P* < 0.05. ^*∗∗*^*P* < 0.01. ^*∗∗∗*^*P* < 0.001 vs. Control group. ^＃^*P* < 0.05. ^＃＃^*P* < 0.01. ^＃＃＃^*P* < 0.001 vs. TGF-*β*1 group.

**Figure 6:** PNS inhibits TGF-*β*1-induced EMT progression through transcription factors snail and TWIST1. The gene and protein of snail and TWIST1 were detected by qPCR and Western blotting, respectively (a)-(b). ^*∗*^*P* < 0.05. ^*∗∗*^*P* < 0.01. ^*∗∗∗*^*P* < 0.001 vs. Control group. ^＃^*P* < 0.05. ^＃＃^*P* < 0.01. ^＃＃＃^*P* < 0.001 vs. TGF-*β*1 group. (c) Then select immunofluorescence technology to further detect the fluorescence expression level of transcription factor snail and TWIST1 (magnification, ×500).

**Figure 7:** The schematic diagram shows how PNS regulates the MAKP and Snail/TWIST1 signaling pathway to inhibit the occurrence of TGF-*β*1-induced EMT.

**Table 1:** Sequence of primers.

Gene	Forward 5′-3′	Reverse 5′-3′
E-cad	GAACACATTTGCCCAATTCCA	ATATAGCTTGAACTGCCGAA
Vim	GGACTCTGATTAAGACGGTT	AGAAAGGCATTGAAAGCTG
FN	TTCCCATTATGCCGTTGGAG	GAAATGACCACTTCCAAAGCCTA
Snail	GGACCCACACTGGCGAGA	AAGGATGTGGGGTCCTTCCT
TWIST1	CGGCCAGGTACATCGACTTC	TCTCTGGAAACAATGACATCTAGG
*β*-actin	ATGACTTAGTTGCGTTACACC	GACTTCCTGTAACAACGCATC

E-cad, E-cadherin; Vim, vimentin; FN, fibronectin.

## Data Availability

Datasets used and/or analyzed in this study can be obtained from the corresponding authors upon reasonable request.
